This article has been retracted.

# Cloud Statistics of Accounting Informatization Based on Statistics Mining

**DOI:** 10.1155/2022/3493678

**Published:** 2022-08-27

**Authors:** Taolan Jin, Bo Zhang, Zhi Yang

**Affiliations:** ^1^School of Economics and Management, Nanjing Vocational University of Industry Technology, Nanjing, Jiangsu 210000, China; ^2^State Grid Taizhou Power Supply Company, Taizhou, Jiangsu 210000, China; ^3^ZTE Nanjing R&D Center, Nanjing, Jiangsu 210000, China

## Abstract

With the rapid development of information technology, the amount of all kinds of data information is increasing rapidly. As an important means to collect, store, and manage massive data, and then analyze and predict the habits and characteristics of certain groups of people and even the development trend of a certain industry, big data technology provides a comprehensive strategic basis for management decision makers that the traditional processing mode cannot match. Contemporary management accounting serves the whole process of enterprise internal control, so it will produce a large number of various data. With the explosive growth of network data and the increasing scale of database, more and more people begin to study data mining, and the classification algorithm, as the key technology in data mining, has also received extensive attention. In order to further improve the information technology level of enterprise management accounting and increase the depth of information application, many enterprises began to pay more attention to data mining, and through deep data mining, the depth and breadth of enterprise data analysis were improved. In the research of data and accounting informatization, data mining technology accounts for about 50% of informatization, which is the way for future development. With the advent of the information age, the dependence of enterprises on information technology in the process of accounting management has been further improved. If enterprises want to achieve better development in the information age, they need to pay more attention to the information technology of management accounting and improve the application ability of enterprise staff in information.

## 1. Introduction

There are many classify algorithms. This study will focus on the decision tree, Bayesian, genetic, artificial neural network, and classify algorithms based on association rules. To construct a management accounting working method system based on statistics mining, we must first make clear the adaptability of statistics mining to management accounting and the central link between statistics mining methods and ideas in management accounting. Statistics mining is an in-depth analysis of the relationship between statistics, finding the relationship between different statistics, then analyzing the business situation of enterprises, finding the problems in business operation, and promoting the overall improvement of financial analysis and decision-making level of enterprises. In statistics analysis technology, statistics classification algorithm has become more and more important. With the deepening of statistics analysis research, more and more statistics classify algorithms have been proposed. A crucial step in statistics classify is to construct a statistics classifier, which is used to accurately classify some unknown types of statistics [1]. In the past, the construction of accounting informatization required the purchase of a large number of hardwares and softwares, and regular maintenance and upgrading also consumed huge costs. Many aspects required a lot of manpower and material support, which increased the operating costs of enterprises. Statistics classify algorithm is the core content of big statistics mining. Its main function is to extract valuable knowledge and message through a large number of operations on massive disordered statistics, analyze the characteristics of all kinds of message, and provide statistics basis for researchers to further predict a certain trend. With the advent of the era of big statistics, the number of statistics that enterprises need to account is also rising, which virtually aggravates the work intensity and difficulty of accountants. As a product of the mature development of the Internet, cloud computing has sufficient network storage space. Cloud computing is a new computing mode based on shared resources, which has developed rapidly in recent years [2, 3]. Cloud storage technology is its core sub-function. Through RAC, networking, or multitiered file storage system, a mass storage device is gathered together through app software to work together, providing convenient and low-cost mass storage services. In the era of big statistics, with the changing development trend of accounting work, the amount of statistics involved in accounting work is increasing, and the difficulty of statistics calculation and analysis is getting higher and higher, which naturally brings great impact to the accounting work of enterprises. Statistics mining is to extract useful knowledge and value from a large number of statistics, which is the inevitable outcome of the development of statisticsbase technology. Statistics mining has been widely used in retail, finance, insurance, medicine, communication, and other fields. Classify is one of the most important technologies in statistics mining, and many algorithms have been proposed so far. Classify is a technology that constructs a classifier according to the characteristics of statistics sets and uses the classifier to assign categories to samples of unknown categories [4].

The goal of accounting is to provide message support for the internal management and control of enterprises. The ultimate goal of the management accounting staff to collect and summarize all kinds of message is to analyze the future production and operation situation of the enterprise based on the past production and operation results, so as to provide support for the strategic decision of the enterprise. The app of statistics mining depends on the message technology of management accounting. Through message technology, the comprehensiveness and depth of statistics can be improved, the financial analysis ability of enterprises can be improved, and the financial management level of enterprises can be improved. With the advent of the statistics era and the development of cloud service technology, the investment in hardware and software in the early stage has been saved to a great extent, and a few computers are often needed, which greatly saves the cost of enterprises. With the wide app of statistics mining technology, statistics classify algorithms are constantly emerging and gradually optimized, among which the classical classify algorithms are decision tree classify algorithm, naive Bayes algorithm, support vector machine classify algorithm, artificial neural network classify algorithm, etc [5].

This study also uses a variety of research methods in its research. In the research of statistics mining, the principle model diagram and algorithm formula are established to study and analyze it. In the research of accounting informatization cloud statistics, the corresponding statistics graph is established to analyze and explain it.

The main contributions of this study are:

1. In this study, an algorithm formula is established to explain the research.
2. In the research of statistics mining in this study, a model diagram is established for analysis.
3. In the research, this study thinks that under the premise of statistics mining, accounting informatization can develop better and better.

The rest of this study is arranged: The second part introduces the related work to make a brief analysis of its research. The third part analyzes and explains the statistics mining. The fourth part analyzes and introduces the accounting informatization. The fifth part summarizes the full text.

## 2. Related Work

As popular technologies such as cloud storage and cloud computing have greatly met the growing demand for storage and computing power, security and privacy issues have become a concern of people. Cloud storage service providers are not completely trustworthy, and the integrity of user statistics may be destroyed due to improper management or insufficient security capability, while bit rot, disk controller error, and tape failure may also cause the integrity of user statistics to be destroyed. Scalability and fast scalability. It can improve the efficiency of accounting when it is applied to the internal accounting work of enterprises. In the process of enterprise management accounting message processing, it is necessary to apply statistics mining technology to carry out statistics analysis, so as to provide reliable statistics support for management accounting, and provide reliable guarantee for the development of enterprises and the improvement of message processing ability. Accounting is a form of accounting work that takes the internal management and control of enterprises as its main service object. Because there is a fundamental difference between financial accounting and financial accounting in the service object, the message that management accounting pays attention to and collects is often not only limited to the single financial message, but also the reflected content is not only the post-reaction and supervision of the enterprise's operating results. Statisticsbase-based knowledge discovery is a computer technology proposed with the rapid development of artificial intelligence and statisticsbase. It searches the hidden useful message from a large amount of statistics by some algorithm, and many fields such as machine learning, pattern recognition, statistics, knowledge acquisition, intelligent statisticsbase, expert system, and high-performance computing are closely related to this technology.

Chen put forward the concept of Merkle Hash Tree, which is a means to greatly reduce the cost of computing hashes for large-scale statistics structures [6]. A short message signature scheme proposed by Hu, Chen, and Ling, compared with RSA and DSA signature schemes, under the same security condition with a modulus of 1024 bits, the BLS signature has a shorter number of signatures [7]. Zheng proposal makes up for the shortage that the Bayesian classify algorithm needs a large number of samples [8]. Shi et al. put forward several improved Bayesian classify algorithms, among which semi-naive Bayesian algorithm, candidate compressed Bayesian network construction algorithm, TAN algorithm, and other effective methods can reduce autonomy [9]. Yunyang et al. proposed a CBA classify method. CBA algorithm is mainly composed of two workflows [10]. Yang proposed a sentinel-based statistics recoverability proof mechanism, which can not only verify the integrity of the statistics on the remote node, but also recover the original statistics to a certain extent if the statistics are damaged [11].

## 3. Research on Statistics Mining Technology

### 3.1. Statistics Mining Technology

The core purpose of statistics mining is to find interesting parts of statistics message, and interpret statistics message from the perspectives of its evolution trend and composition mode. Statistics mining is a key step in knowledge discovery based on statisticsbase, and the knowledge learning stage is usually called statistics mining. For continuous attributes, when each internal node searches for its optimal splitting standard, it is necessary to sort the training set according to the value of the attribute, and sorting is a waste of time. Decision tree classify is an inductive learning method, which predicts a group of random and disordered sample statistics in a tree structure. Decision tree classify algorithm can intuitively reflect the problems and key problems encountered by decision-making classes in each decision-making stage, and is composed of root nodes, internal nodes, leaf nodes, and directed edge nodes. At present, the classical classify algorithms in the stage of big statistics analysis and statistics mining mainly include decision tree, naive Bayes, support vector machine, neural network classify algorithm, and so on. Among the decision tree classify algorithms, the non-C4.5 algorithm is typical, but with the development of computer technology and message technology, 4C5 algorithm can't meet the increasingly complex statistics classify algorithms. Therefore, in order to adapt to the processing of large-scale statistics sets, different classify methods have their own characteristics, and the problems that need to be dealt with are not the same [12]. SL IQ algorithm adopts pre-sorting technology to eliminate the need of sorting statistics sets at each node of decision tree. Decision tree classify algorithm is one of the inductive learning algorithms, which mainly refers to the classify rules that infer “tree” structure from a series of irregular and unordered sample statistics message to predict. Compared with traditional statistics classify algorithms such as statistical methods and neural network methods, decision tree classify algorithm has many obvious advantages. For example, the statistics classify rules of decision tree classify algorithm are simple and clear, easy to understand, and difficult to make mistakes in actual operation. By analyzing and summarizing case sets, the decision tree has the ability of multi-concept learning, which is easy to use and has a wide range of apps [13, 14]. Decision tree algorithm is a better choice when classifying large-scale case statistics represented by unstructured attribute-value pairs. At present, ID3, C4.5, SLIQ and SPRINT are the most commonly used decision tree learning algorithms. In the research, the corresponding model diagrams are established to analyze and explain them, as shown in Figures 1 and 2.

The data mining principle model diagram in Figure 1 further illustrates the application principle of its data mining, and also guides the research of its data mining algorithm. Big statistics mining technology is mainly a process of collecting and dividing statistics messages from massive message statistics according to a specified attribute, and gradually acquiring and accumulating some effective message. As the product of the development of network message technology in the era of big statistics, statistics mining technology mainly involves artificial intelligence, statisticsbase, statistics, and so on. In cloud storage, the schemes for verifying statistics integrity can be divided into statistics holding proof mechanism and statistics recoverability proof mechanism according to whether fault-tolerant preprocessing is applied to the statistics. According to the specific research of classify algorithm, the correlation between the effectiveness of classify algorithm and the characteristics of statistics is strong, and the statistics have vacancy value, loud noise, and dispersion. Part of the statistics has continuous attribute characteristics; Some statistics are scattered and mixed. The process of classifier construction is generally divided into two steps: training and testing. In the training stage, the characteristics of the training statistics set are analyzed, and an accurate description or model of the corresponding statistics set is generated for each category. In the test phase, the test is classified by using the description or model of the category, and its classify accuracy is tested. Generally, the cost of the testing phase is much lower than that of the training phase [15, 16]. Big statistics, as an abstract concept, is simply the mining and integration of massive statistics message. These statistics types are diverse, the statistics volume is huge, the value density is low, and the growth rate is fast. Only by reasonable statistics mining and statistical analysis can the app value behind them be discovered. With the development of production in various industries, a large amount of statistics will be produced every day. Through big statistics technology, this message has a subtle influence on people's current life and even the development of a certain industry.

### 3.2. Research on Statistics Mining Algorithm

The decision tree classify algorithm can intuitively show the problems and key points of decision-making classes in different periods in the whole decision-making process. The decision tree consists of root nodes, internal nodes, leaf nodes, and directed edges connecting nodes. The root node is unique, it represents a group of classified samples, while the internal group represents the attribute of the object, while the terminal node represents the result of the classify. The algorithm starts from the root node, selects the corresponding attribute value from top to bottom, sends the branch to the corresponding node, and repeats this step until the final node and category of the path are stored in the leaf node. Each branch of the decision tree corresponds to a classify rule, so the decision tree classify algorithm can finally output an easy-to-understand rule set. Although the decision tree statistics classify algorithm has many advantages, it also has many disadvantages. Because the decision tree determines the statistics analysis process, in the process of statistics classify, especially in the process of tree construction, it is inevitable to scan and sort the statistics several times in sequence, which will inevitably lead to the whole statistics analysis process becomes slow. Bayes classify algorithm is put forward based on the Bayes formula, and it is an algorithm that uses the knowledge of probability statistics to classify. When the prior probability and class conditional probability are known, the classify algorithm calculates the probability that a given sample with unknown class belongs to each class by Bayes theorem, and selects the class with the highest probability as the determined class of the sample. Li algorithm is improved in many aspects based on 4C5 algorithm technology, and it also adopts sorting technology and breadth-first strategy technology, which makes SLIQ algorithm technology have good scalability for increasing the number of records and attributes to a certain extent. In the research algorithm, corresponding calculation formulas are established to analyze them, such as formulas (1)–(5).

(1) $$\begin{array}{c} 1^{3}\left(-\bar{\Gamma }\right)N=\left\{\begin{array}{c} 1^{7}\left(X\right)Yk_{\Gamma }\left(\begin{array}{c} l_{-}\\ 1 \end{array}\right) \end{array}\right., \end{array}$$

(2) $$\begin{array}{c} \underset{J}{\cap }=c_{i_{\infty }^{1^{1-\infty }-x}\left(y\overset{11}{\underset{t=0}{\prod }}1\right),x_{t}\left|y\right|}, \end{array}$$

(3) $$\begin{array}{c} P_{\left({\text{i}}^{c}|u\right)\infty p{\left(1t\right)}_{a-1}^{\Pi p}C}^{m}x^{41c/3}, \end{array}$$

(4) $$\begin{array}{c} D^{n}{\left(1,11,1L\ldots 1k,\left(J=pkc\right)\frac{1}{1!}\right)}^{1}, \end{array}$$

(5) $$\begin{array}{c} n_{C}=\underset{\partial \varphi }{\text{Res}}\cdot 3\beta Q_{-}^{2+2^{\beta }}Q+\beta . \end{array}$$

Because of the characteristics of C45 algorithm, the structure of decision tree is completed according to the depth-first strategy, so every key node must be analyzed in the process of statistics classify and analysis, and the efficiency is extremely low [17, 18]. However, after the breadth-first strategy technology is adopted, it is only necessary to scan each attribute list once for each layer, and the optimal splitting criteria can be found for each leaf node in the current decision tree. The naive Bayesian algorithm is relatively stable, and it will not have a great impact on the classify results because of the different characteristics of the statistics itself. The stronger the independence between naive Bayesian statistics, the more accurate the classify results. However, we need to pay attention to the premise that the classify algorithm needs to be based on the conditional independence hypothesis, which is an ideal state. In practical app, there will be links between statistics attributes, which will reduce the classify accuracy, so the effect of this method is often difficult to reach the theoretical maximum. It is to improve the ability of statistics processing and increase the value of statistics. From a technical point of view, the relationship between big statistics and cloud computing is inseparable like the front and back of a coin. The existence of big statistics can't be handled by a single computer, so it must be implemented in a multitiered architecture, and massive statistics can be mined in a multitiered way. However, it must rely on cloud computing's multitiered processing and cloud storage virtualization technology. With the advent of the cloud era, big statistics has gradually gained more attention.

SPRIN algorithm has made corresponding changes to the statistics analysis structure of decision tree algorithm, especially deleting the list of statistics categories that need to be stored in memory in SLI *Q* algorithm, and instead merging the list of statistics categories into the attribute list of each statistics number. The advantage of this method is that when analyzing a large number of statistics, it can avoid repeated statistics analysis when traversing each attribute list to find the optimal splitting standard of the current node. In the process of building a decision tree, the most time-consuming operations are the statistical calculation of the category distribution message of the statistics set belonging to each non-terminal node and the splitting of the statistics set by using splitting criteria. Both operations are realized by UDF in *M* IND. Genetic algorithm is an efficient search and random optimization algorithm that evolved from the theory of biological evolution. It is an important breakthrough in the combination of natural science and computer algorithm. With the help of the principle of natural evolution, the algorithm transforms the process of solving problems into the process of finding chromosomes with high fitness according to the genes on chromosomes. This algorithm combines the advantages of directional search and random search, so it has good global search ability, and avoids the disadvantage that most optimization methods are easy to fall into local optimum. The algorithm combines random search with directional search, which makes it have better global optimization performance, and overcomes the defect that the traditional optimal solution is difficult to achieve local optimization [19–21]. Like nature, genetic algorithms can solve problems without knowing them. Its main job is to evaluate all the chromosomes generated in the algorithm, and select the corresponding chromosomes according to their fitness, so that the chromosomes are easier to reproduce. Although the rise of statistics mining research is initiated by researchers in the field of statisticsbase, most of the algorithms proposed so far have not made use of the related technologies of statisticsbase, and it is difficult for statistics mining apps to integrate with statisticsbase systems. This problem has become one of the key issues in this field. In the research of its algorithms, we have once again established its algorithm formulas to analyze and explain them, such as formulas(6)–(9).

(6) $$\begin{array}{c} TC_{u}{\bar{\text{i}}}_{-}^{\sigma -1^{\beta }X_{1}-{\mathbb{R}}_{2}+J_{31}x\prime }, \end{array}$$

(7) $$\begin{array}{c} TS\Sigma_{K+\zeta }^{\prime }:T_{.11}^{L}=5JK_{11}, \end{array}$$

(8) $$\begin{array}{c} -{\bar{l}|}_{1}^{y}x=4tg_{1}\lambda_{1}f\delta {\text{i}}^{x_{2}+\cdots \cdot }+\mu_{2}, \end{array}$$

(9) $$\begin{array}{c} n_{C,x}=\frac{1^{r/2}}{1}=\text{i}\cdot T\ker\phi . \end{array}$$

MIND uses the typical decision tree construction method to build the classifier. The specific steps are similar to SLIQ. The main difference is that it uses the UDF method and SQL statement provided by statisticsbase to construct the tree. Simply put, at each level of the tree, a dimension table is established for each attribute, and the number of each value of each attribute belonging to each category and the node number to which it belongs are stored. CBA algorithm mainly constructs classifier by finding association rules in training set. The classical algorithm Aprio ri is used to discover association rules, which is effective for discovering association rules hidden in a large number of transaction records. At the same time, statistics mining does not artificially limit and exclude the types of statistics to be analyzed. Whether it is financial statistics or non-financial statistics that can be analyzed by accounting subjects, or even non-statistics message, statistics mining does not exclude it. Therefore, statistics mining has strong adaptability to management accounting in two aspects: purpose and object. The method of statistics mining can determine the correlation among all kinds of message through the parameter estimation results of regression analysis, multi-factor variance analysis, and other methods, thus making it possible to identify the influencing factors of the message that managers care about. Genetic algorithm doesn't need to know something about the problem when solving it. Its task is only to evaluate all chromosomes produced in the process of algorithm, and then to screen chromosomes according to the fitness value, among which chromosomes with high fitness value have a greater chance of reproducing the next generation [22–24].

## 4. Research on Accounting Message Statistics

### 4.1. Statistics Mining Management Accounting Message Processing Research

With the development of message technology, financial sharing has good technical conditions. The development of the Internet can realize the sharing of enterprise financial statistics, which has a positive impact on improving the timeliness of financial statistics in enterprise accounting message systems. Cloud computing is an important part of multitiered computing. Specifically, it decomposes huge statistics computing and processing programs into countless small programs, and then processes and analyzes them through a system composed of multiple servers, and feeds back the results of the small programs to users. In the early days of cloud computing, it was also a simple multitiered computing task distribution and integrated computing results. Message management cannot be separated from advanced software and hardware facilities. Therefore, we should first strengthen the construction and improvement of basic management facilities, transform the existing library resources in the library into digital message content through the professional library materials input program, and upload it to the designated library resources platform, so that people can quickly search and download it on the platform. In the message platform, the financial statistics of each region of the enterprise is comprehensively managed, so that the financial statistics can appear on the financial sharing platform in time after it happens, so that the financial personnel can handle the accounts in time after obtaining the relevant statistics, which plays a positive role in improving the timeliness of the financial statistics message in the enterprise accounting message system. In the process of applying the management accounting message system, we should further expand the scope of message processing, help enterprises realize the overall “messagization”, and incorporate the operation statistics of other departments into the accounting message system, so as to realize the supervision and management of the whole enterprise and improve the management effect of the accounting message system. In the research, statistics graphs are established for analysis and interpretation, as shown in Figures 3 and 4.

According to the survey, although some libraries have introduced advanced library message management equipment and set up related intelligent message management platforms at this stage, due to the huge number of books and materials in their collections, there is a problem that the reform of message management mode is incomplete, and most of the books and materials in their collections are still not entered into the message management platform, but kept in traditional paper books. At present, the development of human society has entered the stage of comprehensive informatization, and batch message processing, rapid message transmission and message sharing have become the keywords of the development of the times. It indicates the coming of the era of big statistics. In the process of installation, testing, and operation of accounting message software, a certain amount of capital investment is also needed, which will test the professional ability of financial staff. In the later stage, it is still necessary to upgrade the equipment maintenance software to promote the smooth operation of accounting message construction. Therefore, the continuous cost consumption will aggravate the burden on enterprises, while the traditional accounting message business process is still relatively complicated. The theoretical basis and ideas that statistics mining relies on the process of message selection and trend analysis come from statistics. Among the collected message, it is one of the core ideas of statistics mining to select samples to guess the characteristics of the population and check whether the observed samples belong to the same category as the known population. During the implementation of enterprise management accounting informatization, it is necessary to ensure the reliability and timeliness of the original statistics in order to dig the statistics message deeply. The timeliness of financial work has a very important impact on the level of work and users of financial reports, and the untimely transmission of original statistics has become an important reason that affects the informatization level of enterprise management accounting. In the research, the corresponding statistics graphs are established for analysis and interpretation, as shown in Figures 5 and 6.

When enterprises carry out management accounting work, in the process of message processing, it is necessary to compare the budget statistics, so as to better discover the problems in operation and carry out financial management by mining the differences between the statistics. Enterprise informatization should be applied to budget management, and the management and control of enterprise financial work should be strengthened according to budget statistics. Management accounting message processing based on statistics mining needs to comprehensively improve the depth and breadth of financial statistics, and ensuring the integrity of statistics is an important condition for developing statistics mining and improving message processing ability. The final result of the statistics mining process will be able to provide a powerful help to the core function of management accounting-forecasting. In the management accounting work, the forecast can be divided into two parts: the forecast of the change scale of the existing situation, the forecast of various risks, and the change probability of other uncertain factors. It promotes the internal and external sharing of resources. In the past message environment, although the enterprise supply chain system can share statistics and messages in many aspects, such as production, sales, and finance, and its limitations are still very obvious. Cloud computing technology includes a series of message, such as financial business warehousing, in the platform, breaking down the barriers between various departments, and making the work message of departments no longer presented in the form of message islands, becoming more open and transparent, and sharing internal resources is also an effective supervision for enterprise accounting message.

### 4.2. Research on Accounting Informatization Strategy

Paying attention to the integration and classify of message is one of the optimization strategies to better promote the development of enterprise accounting informatization by using cloud computing technology in the era of big statistics. According to the above analysis, in the current era, the accounting work of enterprises is already facing a huge amount of message, and it is undoubtedly a huge challenge for accountants to complete the processing and processing of various statistics message in a fixed time. Therefore, it is even more necessary to use advanced message technology to classify and sort out the limited financial accounting message inside enterprises and reduce the statistics risks outside enterprises. In order to complete the message collection, analysis, and calculation more conveniently, it is necessary to use the message platform and cloud computing technology to create a more comprehensive and rich enterprise accounting message. In the process of perfecting the management system and system, we can't ignore the improvement of the comprehensive quality of the library management team. First, it is necessary to improve the professional skills of relevant staff, so as to ensure that every staff involved in message management of books and materials can master the operation methods of infrastructure, understand the functions and functions of message management system, and correctly realize the important significance of message management for the management of books and materials. The core function of accounting lies in the supervision and feedback of the existing work results of each process of enterprise management, and the prediction of the long-term changes in enterprise management. In this context, the role of statistics mining will be greatly strengthened. For the management accounting analysis of certain messages, the main functions of statistics mining are cost change analysis, activity-based value analysis, market forecast, and market segmentation. In the research, a statistics map is established to analyze and explain it, as shown in Figure 7.

The management decision of accounting informatization in Figure 7 accounts for about 90% of the whole accounting informatization. Budget is an important part of enterprise's prior management, and it plays a positive role in improving management accounting message processing ability and operation ability. Therefore, in the process of management accounting message processing based on statistics mining, enterprises should incorporate the budget work into the accounting message system of enterprises, use accounting software to analyze the business situation of enterprises, formulate a scientific and reasonable budget in combination with the future development strategy of enterprises, improve the budget management level of enterprises, and narrow the difference between budget and actual statistics. As a manager, you should keep abreast of the development of your own industry and related industries, update your ideas in time, and know the latest trends. In the era of big statistics, the better app of cloud computing technology to the internal financial and accounting management of enterprises needs to improve relevant laws and regulations to ensure the message security. Facing the general trend of message management, we should dare to try, dare to break the traditional model in the past, pay attention to the development of technology and personnel, and realize the development of accounting messages.

## 5. Summary

In the era of big statistics, the emergence of cloud computing technology has brought more possibilities for enterprise accounting informatization, but at the same time, a series of risks still exist. How to seize the opportunity to deal with risks and challenges is still an important problem that every enterprise is facing in the era of big statistics. Systematically studying the classify algorithm of statistics mining will help us to know the advantages and disadvantages of the decision tree classify algorithm, naive Bayes classify algorithm, support vector machine classify algorithm and neural network classify algorithm, as well as their applicable scenarios, and make targeted optimization and improvement on their shortcomings. Big statistics technology and cloud computing technology bring a lot of convenience to the development of accounting informatization, which not only reduces the cost and improves efficiency, but also realizes the sharing of resources, and has great development prospects. With the advent of the era of big statistics, the importance of statistics classify algorithm will become more and more obvious, and the characteristics of algorithms such as execution speed, scalability, and intelligibility of output results will become the trend of statistical analysis. In the process of applying statistics mining to management accounting message processing, enterprises need to pay more attention to the level of financial personnel, improve the level of financial informatization, and provide a human resource foundation for better development of financial informatization.

## Figures and Tables

**Figure 1:** Model diagram of statistics mining sorting principle.

**Figure 2:** Statistics mining classify decision analysis model diagram.

**Figure 3:** Message statistics analysis statistics diagram.

**Figure 4:** Message statistics accounting management analysis diagram.

**Figure 5:** Statistics map of management accounting informatization (1).

**Figure 6:** Statistics map of management accounting informatization (2).

**Figure 7:** Statistics map of accounting message management decision-making.

## Data Availability

The figures used to support the findings of this study are included in the article.
